The article "Application Value of Serum Hcy, TLR4, and CRP in the Diagnosis of Cerebral Small Vessel Disease" was retracted in 2023. Reasons: signs of a paper mill; compromised peer review; unreliable results or conclusions.

# Application Value of Serum Hcy, TLR4, and CRP in the Diagnosis of Cerebral Small Vessel Disease

**DOI:** 10.1155/2022/4025965

**Published:** 2022-04-23

**Authors:** Peng Qu, Kaili Cheng, Qi Gao, Yan Li, Minghua Wang

**Affiliations:** Department of Neurology, The Fifth Affiliated Hospital of Harbin Medical University, Harbin, China

## Abstract

**Objective:**

To evaluate the application value of combined detection of serum homocysteine (Hcy), Toll-like receptor 4 (TLR4), and C-reactive protein (CRP) in the diagnosis of cerebral small vessel disease (CSVD).

**Methods:**

90 patients with CSVD admitted to our hospital within the past year were identified as the research subjects, and the patients with cognitive dysfunction were assigned to the experimental group, and those with normal cognitive function were assigned to the control group according to the evaluation of cognitive dysfunction by the Montreal Cognitive Assessment (MoCA), with 45 cases in each group.

**Results:**

The experimental group obtained remarkably elevated Hcy levels than the control group (*P* < 0.05). The patient's cognitive dysfunction is mainly attributed to the impact of serum Hcy. TLR4 and Hcy were negatively correlated with MoCA scores (*P* > 0.05). In comparison with the control group, the experimental group had significantly higher levels of Hcy, serum CRP, and interleukin (IL)-6 (*P* < 0.05).

**Conclusion:**

The combined detection of serum Hcy, TLR4, and CRP features a high clinical value in the diagnosis of CSVD, which contributes to the prevention and treatment of cognitive dysfunction in patients.

## 1. Introduction

Cerebral small vessel disease (CSVD) refers to a series of clinical, influential, and pathological syndromes that trigger brain white matter and deep gray matter damage due to intracranial small vessel disease, with the pathological changes including loss of smooth muscle cells in the vessel wall, lumen stenosis, thickening of the vessel wall, and precipitation of amyloid. Arteriosclerosis is the main mechanism leading to the pathogenesis of CSVD, which refers to the pathological and physiological changes in the cerebral cortex and medulla after damages to the blood supply through cerebral arterioles and capillaries. As an important subtype of vascular cognitive impairment (VCI), cognitive impairment (CI) triggered by CSVD accounts for about 65% of VCI, which may persistently impair the cognitive and living abilities of patients, seriously compromising the quality of life of patients [1–3]. Homocysteine (Hcy) is closely related to vascular myopathy and is considered an independent risk factor for atherosclerosis. As a free radical scavenger and antioxidant, uric acid is a risk factor for periarterial sclerosis and poses a serious threat to the health of elderly people. TLR4 and C-reactive protein (CRP) are important inflammatory molecules and proteins that participate in the body's natural immunity. They can recognize Gram-negative bacteria lipopolysaccharide (LPS) and heat-shock proteins (HSP) released by host necrotic cells, and the cascade activation reaction of hyaluronate and heparin sulfate-degraded polysaccharides and local endogenous enzymes in the body can also activate TLR4 [4–6]. A common feature of inflammatory or immune-mediated CSVD is cerebral small vessel injury in the context of local or overall inflammation of the organism, and there is a strong correlation between CRP and cerebral microhemorrhages common in CSVD [7]. Accordingly, this study aimed to evaluate the application value of combined detection of serum Hcy, TLR4, and CRP in the diagnosis of CSVD. The report is as follows.

## 2. Materials and Methods

### 2.1. General Information

We identified 90 patients with CSVD admitted to our hospital within the past year as the research subjects and assigned the patients with cognitive dysfunction to the experimental group and the patients with normal cognitive function to the control group according to the evaluation of cognitive dysfunction by the Montreal Cognitive Assessment (MoCA) [7], with 45 cases in each group. The studies involving human participants were reviewed and approved by the Fifth Affiliated Hospital of Harbin Medical University, No. HMU977071.

### 2.2. Inclusion Criteria

The inclusion criteria were as follows: all patients met the diagnostic criteria for CSVD in the “Consensus on the Diagnosis and Treatment of Cerebral Small Vascular Disease” [8]. Diagnostic criteria were as follows: de novo small focal cerebral infarcts, lacunae, cerebral white matter high signal, microhemorrhage, and perivascular gaps are the main imaging changes in cerebral small vessel disease. The above imaging changes increase significantly with age, with complete clinical data, and the patients and their families signed the informed consent form after being fully informed of the purpose and process of the study.

### 2.3. Exclusion Criteria

The exclusion criteria were as follows: patients with recent use of drugs that can affect the Hcy level; with head trauma, encephalitis, and thyroid dysfunction that impair cognitive function, or with dementia; with serious medical diseases such as respiratory failure, severe renal insufficiency, acute heart failure, and tumor; with severe audiovisual dyslexia and inabilities to cooperate the research; and with incomplete clinical data.

### 2.4. Methods

The general information of the patients was collected.

In the early morning of the second day after admission, 5 ml of peripheral venous blood was collected from the patients, and the Hcy level was determined by the circulating enzyme method. The operation strictly complied with the instructions of the kit during the test.

TLR4, CRP, and interleukin (IL)-6 were determined by enzyme-linked immunosorbent assay (ELISA, Abcam, ab22048; ab18039; and ab233706), with the reference of TLR4 ≤9.7 mIU/ml. The TLR4 kits were provided by Shanghai Yubo Biotechnology Co., Ltd.

### 2.5. Observational Indicators

The Montreal Cognitive Assessment (MoCA) was used to evaluate the cognitive functions of patients, including space, execution ability, attention, calculation ability, and abstract thinking, with 30 minutes as each measurement interval.

### 2.6. Statistical Analyses

The data processing software selected in this research was SPSS 20.0, and GraphPad Prism 7 (GraphPad Software, San Diego, USA) was used to plot the graphics. The counting data adopted the *X*^2^ test and was expressed by (*n* (%)), and the measurement data were expressed by $\left(\bar{x}\pm s\right)$ and analyzed by the *t*-test. *P* < 0.05 indicates that the difference is statistically significant.

## 3. Results

### 3.1. A Univariate Analysis of Factors Affecting Cognitive Function in Patients with CSVD

The two groups presented no great disparity in terms of the general information including age, gender, BMI, course of the disease, smoking, drinking, and place of residence (*P* > 0.05), as given in Table 1.

### 3.2. MoCA Scores

Significant differences were found in the MoCA scores between the two groups of patients (*P* < 0.05), as given in Table 2.

### 3.3. Correlation between Serum TLR4, Hcy, and Mild Cognitive Impairment in CSVD

There was a negative correlation between serum TLR4, Hcy, and MoCA scores (*P* > 0.05), as given in Table 3.

### 3.4. Multivariate Logistic Regression Analysis of Influencing Factors

Logistic regression analysis indicated that Hcy, TLR4, and age correlated with the cognitive function of CSVD patients (*P* < 0.05), as given in Table 4.

### 3.5. Serum Indexes

The levels of serum CRP and interleukin (IL)-6 in the experimental group were significantly higher than those in the control group (*P* < 0.05), as shown in Figure 1.

## 4. Discussion

CSVD is one of the common diseases in clinical practice to which elderly populations are more susceptible. It poses a serious threat to the health and safety of patients, compromises the quality of life of patients, and poses a huge burden to the patients' families and society. There are still many unknown areas in clinical research on CSVD currently, and the relationship between CSVD and related clinical manifestations is elusive [9–12].

Hcy is a metabolite of methionine produced by the methylation reaction in the liver and the kidney, for which methionine cycle and transsulfide are the main metabolic pathways, and the deficiency of cofactors and enzymes in each metabolic pathway may result in the increase of Hcy levels. Previous studies have proposed that a high level of Hcy damage cerebrovascular or causes neuro virus, a high level of Hcy ultimately damage the endothelial function by mitigating the endothelium-dependent vasodilation reaction and inhibiting the immune activity of nitric oxide synthase, which gives rise to the shedding-off of endothelial cells and the aggregation of platelet around the wound of the vascular wall, and eventually generates thrombus [13–16], and a high level of Hcy can thicken the growth of vascular smooth muscle and increase the thickness of the vascular intima-media, thereby damaging the blood vessels. Therefore, a high level of Hcy is associated with cerebral arteriosclerosis, brain atrophy, and ischemic necrosis, which will eventually result in cognitive dysfunction in patients. TLR4 is an important inflammatory molecule involved in the body's natural immunity and a key substance that connects natural immunity and specific immunity [16–21].

Prior research has pointed out that Hcy is related to the degree of cognitive function of patients with CSVD; moreover, serum Hcy compromises patients' cognitive functions and hinders the executive ability and attention of patients with CSVD [22, 23]. Research by Ito et al. [23] showed that impaired vascular endothelial cell function is the main cause of CSVD. Furthermore, the research results by de la Cruz-Cosme et al. [24] have demonstrated that high Hcy levels are related to cognitive impairment and the degree of cognitive impairment. The research has shown that Hcy damages vascular endothelial cells through the interaction with thrombomodulin and tissue factor pathway grafts and participates in the occurrence and development of cognitive dysfunction in patients with CSVD [24]. Currently, many different biological mechanisms can associate high levels of Hcy with cognitive dysfunction, including vascular mechanisms, regional brain atrophy, neurofibrillary tangles, amyloid plaque formation, neuronal death, and epigenetics mechanism. Similar to several studies, neurological damage and blood-brain barrier disruption after CSVD lead to the release of proteins in the brain, which can be recognized by the body as “heterologous” antigens. These antigens will activate innate immune cells that reside in the CNS to stimulate cytokine release, thus promoting the differentiation and expansion of antigen-specific T cells, leading to a cellular immune response, and possibly activating B cells to generate a humoral immune response [20, 21]. Collectively, these immune responses lead to neuronal and glial cell damage in CSVD. Consistent with other etiologies of CSVD, immune and inflammation-mediated CSVD can manifest clinically with cognitive decline and dementia, neuropsychiatric symptoms (including hallucinations, agitation, depression, anxiety, apathy, irritability, sleep disturbances, and appetite changes), urinary symptoms (including nocturia, incontinence, urinary frequency, and urgency), and gait disorder symptoms (including impaired motor and balance). Through the treatment and observation of massive CSVCI cases, TCM believes that this disease is attributable to the phlegm and dampness, stagnation of blood, and obstruction of orifices due to deficiency of kidney essence and internal depletion of essence and blood. The basic pathogenesis is the deficiency of the medulla oblongata and loss of use of the divine mechanism, whereby the causative factors can be summarized as “deficiency, phlegm, and stasis.” Patients with CSVD are mostly accompanied by urinary incontinence and abnormal gait, which is due to old age, physical weakness, deficiency of kidney Qi, loss of bladder, and lack of solidity of the lower energy, resulting in incontinence of urine. After years of experience, a formula of Naosuikang (Astragalus, *Pueraria mirifica*, Radix et Rhizoma Ligustici, Rhizoma Ligustici, Radix *Salvia miltiorrhiza*, Rhizoma Tenuifolia, Radix Scorpion, Cornu Cervi Pantotrichum, Radix *Angelica sinensis*, and Radix et Rhizoma Polygonati) was developed for the treatment of this disease with remarkable efficacy. *Eucommia*, *Achyranthes bidentata*, and *Fructus lycii* were added for back pain and leg weakness, *Acorus calamus*, *Fructus hallucinogens*, and *Poria cocos* were added for phlegm obstruction, *Guadua piperita*, Zhushu, and Zhaobei mum were added for phlegm-heat, peach kernel, safflower, and chicken blood vine were added for blood stasis obstruction, and hooked vine and oyster were added for rheumatism.

## 5. Conclusion

Both low HDL and high Hcy may trigger cognitive dysfunction in patients with CSVD, the detection of which contributes to improving patients' cognitive dysfunction.

## Figures and Tables

**Figure 1:** Comparison of serum indexes between the two groups of patients. The abscissa represents the diagnosis, and the ordinate represents the serum index. The CRP and IL-6 of the experimental group after diagnosis were (9.96 ± 1.54) mg/L, (1.11 ± 0.28) ug/L, and (15.67 ± 3.81) pg/mL, respectively. The CRP and IL-6 of the control group after diagnosis were (7.09 ± 1.28) mg/L, (0.05 ± 0.02) ug/L, and (8.52 ± 2.39) pg/mL, respectively. ^*∗*^There is a significant difference in CRP after diagnosis between the two groups (*t* = 10.134, *P* < 0.05). ^*∗∗*^There is a significant difference in IL-6 between the two groups of patients after diagnosis (*t* = 13.698, *P* < 0.05).

**Table 1:** A univariate analysis of factors affecting cognitive function in patients with CSVD (*n* (%)).

	Experimental group (*n* = 45)	Control group (*n* = 45)	*x* ^2^ or *t*	*P*
Age (year)	46.75 ± 3.32	46.69 ± 3.29	0.086	>0.05
Gender				
Male	23 (51.11)	21 (46.67)	0.178	>0.05
Female	22 (48.89)	24 (53.33)		
BMI (kg/m^2^)	26.27 ± 1.59	25.89 ± 1.63	1.119	>0.05
Hypertension	21 (46.67)	26 (57.78)	1.113	>0.05
Diabetes	6 (13.33)	10 (22.22)	1.216	>0.05
Coronary heart disease	1 (2.22)	4 (8.89)	1.906	>0.05
Smoking				
Yes	20 (44.44)	21 (46.67)	0.045	>0.05
No	25 (55.56)	24 (53.33)		
Drinking				
Yes	22 (48.89)	24 (53.33)	0.178	>0.05
No	23 (51.11)	21 (46.67)		
Place of residence				
Urban	31 (68.89)	30 (66.67)	0.050	>0.05
Rural	14 (31.11)	15 (33.33)		

**Table 2:** Comparison of MoCA scores between the two groups.

Groups	Experimental group	Control group	*P*	*t*
Visual space and execution ability	2.98 ± 1.34	4.29 ± 0.84	<0.05	5.557
Naming	2.67 ± 0.43	2.84 ± 0.24	<0.05	2.316
Attention	3.54 ± 1.08	5.17 ± 0.83	<0.05	8.028
Language	1.83 ± 0.76	2.29 ± 0.63	<0.05	3.126
Abstract thinking	1.38 ± 0.66	1.79 ± 0.41	<0.05	3.540
Delayed memory	3.23 ± 1.06	3.76 ± 0.83	<0.05	2.641
Orientation	5.28 ± 0.94	5.86 ± 0.37	<0.05	3.851
MoCA scores	21.03 ± 3.19	27.13 ± 1.12	<0.05	12.103

**Table 3:** Correlation between serum TLR4, Hcy, and mild cognitive impairment in CSVD.

Indicators	TLR4		Hcy	
	*r* value	*P* value	*r* value	*P* value
MoCA scores	−0.314	0.007	−0.441	<0.01
Visual space and execution ability	−0.427	0.006	−0.362	0.002
Naming	−0.459	0.004	−0.033	0.071
Attention	−0.411	0.005	−0.093	0.273
Language	−0.014	0.596	−0.394	0.006
Abstract thinking	−0.372	0.025	−0.062	0.356
Delayed memory	−0.081	0.322	−0.271	0.023
Orientation	−0.039	0.421	−0.116	0.941

**Table 4:** Multivariate logistic regression analysis of influencing factors.

Groups	B value	SE	Wald value	OR value	95% CI	*P* value
Age	−0.105	0.035	7.664	0.894	0.821–0.974	<0.01
Coronary heart disease	−0.972	0.675	2.072	0.384	0.098–1.426	>0.05
Diabetes	−0.621	0.557	11.263	0.534	0.179–1.593	>0.05
Hypertension	−0.479	0.284	2.347	0.621	0.361–1.069	>0.05
Hcy	−0.322	0.053	31.653	0.725	0.652–0.801	<0.01

## Data Availability

No data were used to support this study.
